RETRACTED

# MS14 Down-regulates Lipocalin2 Expression in Spinal Cord Tissue in an Animal Model of Multiple Sclerosis in female C57BL/6

**DOI:** 10.6091/ibj.1375.2014

**Published:** 2014-10

**Authors:** Abbas Ebrahimi-Kalan, Jafar Soleimani Rad, Laya Kafami, Daryoush Mohammadnejad, Mehryar Habibi Roudkenar, Amir Afshin Khaki, Zeynab Aliyari, Amaneh Mohammadi Roushandeh

**Affiliations:** 1 *Dept. of Neurosciences, School of Advanced Medical Sciences, Tabriz University of Medical Sciences, Tabriz, Iran;*; 2 * Shefa Neuroscience Research Center, Tehran, Iran;*; 3 * Dept. of Pathobiology, School of Medicine, Alborz University of Medical Sciences, Karaj, Iran; *; 4 *Blood Transfusion Research Center, High Institute for Research and Education in Transfusion Medicine, Tehran, Iran; *; 5 *Dept. of Anatomical Sciences, School of Medicine, Hamadan University of Medical Sciences, Hamadan, Iran*

**Keywords:** Lipocalin2 (LCN2), MS14, Experimental autoimmune encephalomyelitis (EAE), Multiple sclerosis

## Abstract

**Background: **Experimental autoimmune encephalomyelitis (EAE) is an animal model of multiple sclerosis, which is a demyelinating and an inﬂammatory disease of central nervous system. Recent studies have established that some molecules such as Lipocaline2 (LCN2), which expresses during inflammatory conditions, play an important role in EAE pathogenesis and might involve in its treatment process. Recently, it has been proved that MS14, an herbal-marine drug, has anti-inflammatory properties through reduction of TNF-α and IL-1β. Thus, the present study investigated the effects of MS14 on the course of EAE and its relation to LCN2 expression in both protein and gene levels. **Methods: **EAE was induced in female C57BL/6 mice using Hooke kits. Animals were scored for clinical signs of the disease according to a 10-point EAE scoring system. On 21^st^ and 35^th^ days after immunization, mice (n = 4/group) were deeply anesthetized, and the spinal cords were removed. Inflammatory cell infiltration and LCN2 expression in spinal cord were assessed by hematoxylin and eosin staining, immuno-histochemistry, and real-time PCR methods. **Results:** MS14 significantly ameliorated EAE symptoms and decreased lymphocyte infiltration into the spinal cord (*P*<0.05). Our data also revealed that LCN2 expression was significantly down-regulated in acute and chronic phases of EAE both at protein and gene levels after MS14 treatment (*P*<0.05). **Conclusion: **The results demonstrated that MS14 regulatory effect on EAE is accompanied by LCN2 down-regulation after treatment with the herb; however, more studies are required for clarifying the other involved mechanisms.

## Introduction

Multiple sclerosis (MS) is an autoimmune demyelinating disease of central nervous system (CNS) in young adults. Neuro-inflammation, which is composed of mononuclear cell infiltration into the CNS through damaged blood brain barrier, is known as an early pathological event occurred in MS [1-3]. Inflammatory mediators and oxidative agents, such as nitric oxide and reactive oxygen species, which are produced by inflammatory cells, result in demyelination and axonal damage [4-7]. Contribution of oxidative stress, which is an imbalance between the free radical level and the antioxidant defense mechanisms, has been demonstrated in neurodegenerative diseases such as MS. Furthermore, the implication of inflammatory processes in MS and its experimental animal model i.e. EAE has been proved [4-9]. Therefore, antioxidant therapy, including herbal drugs, is of great interest in MS treatment.

RETRACTED

MS14 an herbal-marine drug has been recently explained. According to analytic data, this compound contains many inorganic salts. It has anti-inflammatory and immunomodulatory effects through reduction of TNF-α and IL-1β production in MS and EAE [10]. Due to these anti-inflamatory effects it is considered as a potential therapy for MS [11, 12]. However, effects of MS14 on oxidative stress and the mechanisms underlying regulates the immune system remain unknown. 

Lipocaline2 (LCN2), which is a member of the lipocalin family of transport proteins and an acute phase of reactive protein, usually is expressed during inflammatory and oxidative stress conditions [13, 14]. LCN2 plays an important role in EAE and is up-regulated during the disease course [15, 16]. 

Strategies employed in MS treatment are based on the reduction of lymphocyte reactivity and the extent of neuroinflammation. Although an immunomodulatory effect of MS14 has been proved, this effect on EAE has not been fully understood. Therefore, the present study was undertaken to investigate the expression of lipocalin2 level as well as the effects of MS14 on the course of EAE and its relation to Lipocalin2 expression. In other words, this study was conducted to determine whether there was any correlation between LCN2 expression and EAE as well as whether the administration of MS14 resulted in any change in the expression level of LCN2.

## MATERIALS AND METHODS

***Animals. ***C57BL/6 female mice (n = 25, 8-10 weeks old) were purchased from Pasture Institute of Iran (Tehran). The animals were housed in a pathogen-free animal condition with standard humidity and 22-23°C temperature and 12/12 (7 AM–7 PM) dark/light cycle. Four animals were housed in each cage and maintained one week for acclimatization and then weighted once a week during the experiment. All the experiments were approved by the Ethical Committee of Tabriz University of Medical Sciences Tabriz, Iran. 

RETRACTED

***Experimental autoimmune encephalomyelitis induction*** **. **Mice were immunized with Hooke kits (Hooke laboratories, EK-0115, Lawrence, MA, USA) according to the manufacturer’s instructions. Briefly, after a mild anesthesia, 0.1 ml MOG_35-55_/CFA emulsion was injected subcutaneously into both flanks of each mouse (0.2 ml/animal). Then, the mice received intraperitoneal injections of pertussis toxin (0.1 ml/animal/day, i.p.) on the same day and 24 hours later. 

***Treatment groups*** **. **Mice were randomly divided into control (n = 13) and MS14-treated (n = 12) groups. All animals were housed separately in each cage with access to food and water *ad libitum*. Animals in treated group received food containing MS14 (30% of food weight) from the day of immunization to the end of the study. MS14 powder was a gift from Pharmacology Department of Shahed University by decedent Dr. Amrollah Ahmadi [12]. 

***Clinical evaluation. ***Animals were evaluated and scored for clinical signs of the disease by a researcher blind to the treatments from day 7 to day 35 post immunization using the 10-point EAE scoring system as follows: 

0, no clinical sign; 0.5, partial tail paralysis; 1.0, complete tail paralysis; 1.5, complete tail paralysis and discrete hind limb weakness; 2.0, complete tail paralysis and strong hind limb weakness; 2.5, unilateral hind limb paralysis; 3, complete hind limb paralysis; 3.5, hind limb paralysis and forelimb weakness; 4.0, complete paralysis (tetraplegia), and 5.0, moribund or dead [17, 18]. The successful induction of EAE in all mice in both groups was confirmed by this scoring scale. Three clinical parameters were analyzed to compare the course of EAE between the two groups: severity of disease with cumulative disease index, which was calculated for each mouse as the sum of the daily clinical scores for the entire duration of disease, disease onset and peak score of the disease, i.e. the highest score reached by each animal during the course of disease [18]. Having the highest clinical signs of disease without any improvement for at least three uninterrupted days was determined as an acute phase. Also, remaining the disease for three continuous days was defined as chronic phase.

***Histopathological analysis. ***After 35 days post immunization, mice were deeply anesthetized with ketamine/xylazine (5/1) and perfused with cold PBS. Half of the tissues was sent for histopathology and put in the 4% paraformaldehyde for 72 h, and another half was labeled and stored at -80ºC for further RNA extraction and gene expression. Spinal cords were removed and immersed in 4% paraformaldehyde for 72 hours. Fixed tissues were paraffin-embedded, and 5-μm sections were prepared from the lumbar spinal cords. The sections were deparaffinized through xylol and stained with hematoxylin and eosin with a routine protocol. Five randomly selected sections of lumbar spinal cord in each animal were scanned and photographed using a light microscope (Axioskop2; Carl Zeiss MicroImaging Inc., Germany). Inflammatory cuff surface in the white matter in each section was measured using INFINITY software (version 4.6.0). 

RETRACTED

***Immuno-histochemistry staining.*** Spinal cord tissues (n = 3/group) were obtained from mice sacrificed on 21^st^ and 35^th^ days after immunization and cryoprotected in 30% sucrose solution at 4°C overnight. Tissue passage was performed routinely, and 5-µm thickness cross sections were prepared using a microtome (Sakura, Japan) and picked up on gelatin-coated slides. After incubation at 58°C overnight, the slides were deparaffinized in xylene and rehydrated in descending alcohol solutions. Then, the sections were blocked in BSA [10% BSA in PBS containing 0.1% Triton X-100 in PBS] and incubated with rabbit anti-mouse LCN2 monoclonal antibody (1:100, Abcam, USA) at 4°C overnight. The sections were then incubated with FITC goat anti-rabbit secondary antibody at 1:500 dilution at room temperature for 1 hour, washed with PBS, and mounted using Fluoromount-G 90% glycerin (Southern Biotech, AL, USA). The slides were visualized with fluorescent microscopy (BX51WI; Olympus, Tokyo, Japan) to detect LCN2 expression.

***RT-PCR and real-time PCR*** **. **RT-PCR and real-time PCR were used to investigate any differences in the expression of LCN2 gene between the groups. Briefly, the spinal cords were removed immediately from euthanized mice on 21^st^ and 35^th^ days after immunization (n = 4/group/time point) and stored at -80°C until RNA extraction. Total RNA was extracted from the samples by Trizol reagent (Invitrogen, Carlsbad, CA, USA) according to the manufacturer’s protocol. cDNA was synthesized from 1 µg of total RNA, followed by DNaseI (Invitrogen, USA) treatment and heat inactivation according to the manufacturer’s protocol (Bioneer, USA). RT-PCR was performed using a commercially available master mix (Amplicon, Germany) in a GeneAmp PCR system 9600 (PerkinElmer Life and Analytical Sciences, Wellesley, MA). After initial denaturation (at 94°C for 5 min), cDNA was subjected to 33 cycles of PCR (at 94°C for 30 s, at 59°C for 30 s, and at 72°C for 30 s) using 5′-CCA GTT CGC CAT GGT ATT TTT C-3′ as a forward primer and 5′-CAC ACT CACCAC CCA TTC AGT T-3′ as reverse one. The expression of β-actin was used as an internal control using 5’-TTC TACAAT GAG CTG CGT GTG G -3’ and 5’-GTG TTGAAG GTC TCA AAC ATG AT-3’ as forward and reverse primers, respectively. PCR products were separated on 2% agarose gel. Real-time PCR was carried out using a Rotor-Gene 3000 system (Corrbet, Germany) with the mentioned primers. Ampliﬁcation was conducted using Takara solute sybr green ROX mix (Takara, Japan) according to the manufacturer’s instruction. Briefly, initial denaturation was adjusted at 94°C for 5 min and followed by 40 ampliﬁcation cycles, consisting of denaturation stage at 94°C for 30 s, annealing stage at 59°C for 30 s, and extension stage at 72°C for 30 s. Threshold cycle values were normalized by β-actin expression.

RETRACTED

***Statistical analysis. ***Clinical signs, inflammation, and LCN2 expression in spinal cord were analyzed using Mann-Whitney test and student’s *t*-test. Values of *P*<0.05 were considered to be statistically significant.

## RESULTS

***MS14-reduced clinical signs of the experimental autoimmune encephalomyelitis***. MS14 significantly decreased the daily clinical score of the disease at effector phase of the disease (*P*<0.05, days 22-35 after immunization, Fig. 1). Cumulative disease index showed MS14-treated animals (36.43 ± 4.8) had lower EAE severity than the control animals (53.25 ± 4.88) (*P*<0.05). The rate of clinical score at chronic phase of the disease (day 30 to 35 after immunization) was significantly lower in MS14-treated group compared to controls (*P*<0.05, Fig. 1). Time to EAE onset was detected approximately on day 12 after immunization and reached to a peak stage on day 21 after immunization, where the most animals remained ill (score 2.5-3) throughout the entire experimental period (35 days after immunization, Fig. 1). MS14 neither affected clinical scores at the peak of the disease nor delayed time to EAE onset significantly. Animals were weighted once a week during the experiment, but there was not observed significantly any difference between the groups.

**Fig. 1:** Effects of MS14 on daily clinical score of EAE during 35 days after immunization. Daily clinical score of MS14-treated group was compared to control group using Mann Whitney test. Values are shown as means ± SEM. MS14 suppressed significantly the signs of the disease from 22 days after immunization to the end (*P<0.05). Open (○) and black circles (●) represent mean daily clinical score for MS14-treated and control groups, respectively. Asterisk shows significant difference

***MS14 suppressed neuroinflammation. ***The inflammatory cell infiltration into spinal cord was evaluated using hematoxylin and eosin staining. The analysis of white matter surface occupied by inflammatory cells compared to whole white matter surface of spinal cord tissue indicated that MS14 treatment significantly decreased the inflammatory plaques in the spinal cord in EAE animals (*P*<0.05, Fig. 2).

RETRACTED

**Fig.2:** Effects of MS14 on inflammatory cell infiltration into spinal cord. Lymphocyte infiltrations in spinal cord have been evaluated by hematoxylin and eosin staining and arrows have been demonstrated lymphocyte infiltration. Infiltrated cells were measured at axial section of spinal cord in control and MS14-treated groups on the 35^th^ day after immunization. Values are shown as mean ± SEM., the infiltrated surface of the spinal cord was signiﬁcantly smaller in MS14-treated (A = 7.08 ± 1.50) than control group (B = 26.70 ± 6.50) group (*P<0.05). Asterisk shows significant difference. Magnification (100 × and 400 ×).

**Fig. 3:** Effects of MS14 on Lipocalin-2 (LCN2) protein induction. LCN2/ neutrophil gelatinase-associated lipocalin was detected in paraformaldehyde-fixed paraffin-embedded sections of spinal cord using monoclonal anti-mouse LCN2 antibody. MS14 treatment attenuates the LCN2 expression **(A)** in comparison with the control group **(B)**.

***MS14 down-regulated LCN2 expression. ***The expression of LCN2 at protein level was determined by immune-histochemical staining. Our findings showed that LCN2 was expressed in both control and MS14-treated groups. Also, LCN2 expression was dramatic-ally decreased in MS14-treated group compared to the control (Fig. 3). To evaluate LCN2 gene expression in spinal cord tissue, RT-PCR and real-time PCR were performed. Semi-quantitative expression of LCN2 was shown in all groups even in a normal mouse without any interference (lane 1, Fig. 4). RT-PCR indicated the alteration of LCN2 gene expression during acute and chronic phases of the disease in control mice. LCN2 was down-regulated in MS14-treated group compared to control in acute phase (lanes 2 and 3, Fig. 4). Similar result was found in chronic phase as well (lanes 4 and 5, Fig. 4), while LCN2 up-regulated at acute phase in both groups. 

**Fig. 4:** Effects of MS14 on LCN2 gene expression. **(A)** LCN2 gene expression determined by RT-PCR in control and MS14 groups at acute and chronic phases. **(A)** Lane 1 (normal), lane 2 (control at acute phase), lane 3 (MS14 at acute phase), lane 4 (control at chronic phase), and lane 5 (MS14 at chronic phase). Up-regulation of LCN2 is shown in acute phase of EAE. **(B)** β-actin expression is shown in all groups. **(C)** Fold changes of LCN2 expression in both control and MS14 groups at acute and chronic phases. The level of LCN2 expression is higher at acute phase and strongly is affected by MS14 at chronic phase (*P<0.05). Asterisks show significant differences. Our results showed a significant decrease in LCN2 expression in MS14-treated group during acute phase (2.65 ± 0.34) compared to control group (5.32 ± 0.37, *P*<0.05). Similar results were shown in control and MS14 groups (4.34 ± 0.29 vs. 1.123 ± 0.17) during chronic phase. M, marker

However, the influence of MS14 at chronic phase was remarkable. LCN2 expression in spinal cord was quantified by real-time PCR performed in both experimental groups. Our results showed a significant decrease in LCN2 expression in MS14-treated group during acute phase (2.65 ± 0.34) compared to the control group (5.32 ± 0.37, *P*<0.05). Similar results were shown in control and MS14 groups (4.34 ± 0.29 vs. 1.123 ± 0.17) during chronic phase. Interestingly, both groups showed a significant decline in LCN2 expression during chronic phase (*P*<0.05, Fig. 5). LCN2 protein and gene were expressed in spinal cord tissue in both experimental groups.

RETRACTED

## DISCUSSION

In this investigation, we report that MS14 has suppressive effects on EAE at effector phase of the disease and reduces inflammatory cell infiltration into CNS. The results of the present study revealed that the expression of LCN2 was down-regulated by MS14 in acute and chronic phases of EAE. 

The suppressive effects of MS14 can be attributed to its anti-inflammatory effects, which have been shown by several studies. These studies indicate that MS14 is able to modify the innate and cellular immune responses [10-12, 19]. MS14 exerts its anti-inflammatory effects through decline in Th1 function and up-regulation of Th2 cytokines such as IL-5 and IL-10, which in turn can** s**uppress inflammation [10, 20]. To support this notion, Tafreshi *et al.* [12] and Aktas *et al.* [21] reported that herbal drugs such as MS14 and green tea had anti-inflammatory effects and resulted in alleviation of EAE. 

Furthermore, our result revealed that MS14 inhibited inflammatory cell infiltration into CNS and protected the nervous tissue from further damages, suggesting the positive effects of MS14 on MS patients [11, 22] might be, at least, due to this function of MS14. 

We also reported that the expression of LCN2 was up-regulated in all stages of EAE, and interestingly after the administration of MS14 the expression was down-regulated. In our investigation, higher expression of LCN2 was considerably observed at acute phase. This result is in agreement with data obtained by Berard *et al.* [15]. They reported that expression of LCN2 is induced in the early stages of EAE. They also found that higher expression of LCN2 can be observed specifically in infiltrated monocytes and astrocytes [15]. 

 Precise role of LCN2 remain unknown so far; however, the implication of LCN2 expression has been reported in several diseases [23, 24]. Antioxidant property is one of the well-known functions of LCN2 [13]. Recently, it has been shown that LCN2 is induced in CNS following lipopolysaccharide administration [25]. Moreover, TNF-α, IL-17 and IL-6 can induce LCN2 expression. On the other hand, the expressions of these pro-inflammatory cytokines have been detected in EAE and MS lesions [15]. Taken together, we believe that due to oxidative stress and inflammatory condition expression of LCN2 is induced and this induction is a compensatory reaction to alleviate the stressful conditions. To support this notion, in this study, following administration of MS14, as an anti-oxidant and anti-inflammatory agent, the expression of LCN2 was down-regulated. 

RETRACTED

However, the role of LCN2 in MS could be even controversial. We know that LCN2 enhances matrix metalloproteinase-9 (MMP9) activity [26]. On the other hand, MMP9 facilitates inflammatory cells infiltration into CNS during MS by destructing blood brain barrier. Together, this suggests contribution of LCN2 in the pathogenesis of MS. In other words, LCN2 may exacerbate the severity of the disease. However, these might be fortunate for intervention which can be modified by some therapeutic approaches. So, as our study revealed MS14 might be pertinent in this regard. 

In summary, our results highlight the importance of LCN2 expression in EAE. The induction of LCN2 in early stages of EAE suggests that LCN2 might be considered as an early biomarker for MS. Our results also indicated that the administration of MS14 not only alleviates the EAE symptoms but also down-regulates LCN2expression. However, the precise role of LCN2 in EAE warrants further and complementary studies. 
